RETRACTED

# Serum Levels of HCY, MIF, and hs-CRP Correlate with Glycolipid Metabolism in Adults with Never-Medicated First-Episode Schizophrenia

**DOI:** 10.1155/2021/7394699

**Published:** 2021-11-13

**Authors:** Xiao Zhong, Qin Ao, Fei Xing

**Affiliations:** ^1^Psychiatry Department, Jiangxi Province Honorary Military Rehabilitation Hospital (Jiangxi Kangning Hospital), Yuhushan Avenue, Xinjian District, Nanchang 330103, Jiangxi Province, China; ^2^Department of Clinical Laboratory, The Second People's Hospital of Huai'an, No. 62, Huaihai South Road, Huai'an City 223001, Jiangsu Province, China

## Abstract

**Objective:**

It has been reported that the prevalence of metabolic syndrome (MS) in multiepisode patients with schizophrenia is 35.3%, which is 2- to 4-fold higher than in the general population. The study is designed to compare the glycolipid metabolism in patients with first-episode schizophrenia (FES) with sex- and age-matched healthy controls to investigate changes in serum levels of homocysteine (Hcy), macrophage migration inhibitory factor (MIF), and high-sensitive C-reactive protein (hs-CRP) and their relationships with the glycolipid metabolism in patients with FES.

**Methods:**

His case-control study included 88 patients diagnosed with FES and 88 sex- and age-matched healthy controls. Patient psychopathology was assessed using the Positive and Negative Syndrome Scale (PANSS), Young Mania Rating Scale (YMRS), and 17-item Hamilton Rating Scale for Depression (HAMD-17). Patients with FES were classified into MS and non-MS groups.

**Results:**

There were significant differences in the education level, body mass index (BMI), and waist circumference between the patients with FES and healthy controls (all *p* > 0.05). The patients with FES had higher levels of FPG and blood glucose at the oral glucose tolerance test (OGTT) (2 h glucose) concomitant with higher proportion of impaired glucose tolerance (IGT) and homeostasis model assessment of insulin resistance (HOMA2-IR) than healthy controls (all *p* < 0.001). It was revealed that the patients with FES showed higher serum levels of Hcy, MIF, and hs-CRP than healthy controls (all *p* < 0.001). The serum level of Hcy shared positive correlations with the score of PANSS totals (*r* = 0.551) and the negative syndrome of the PANSS scale (*r* = 0.494). The serum levels of MIF and hs-CRP was only positively correlated with the negative syndrome of the PANSS scale (*r* = 0.320 and *r* = 0.446). The level of Hcy shared positive correlations with the levels of FPG, 2 h glucose, and HOMA2-IR; the level of MIF was only positively correlated with the level of HOMA2-IR; the level of hs-CRP had a positive correlation with both levels of FPG and 2 h glucose (all *p* < 0.001). The levels of Hcy, MIF, and hs-CRP all shared positive correlations with the TG level and negative correlations with the HDL-C level (all *p* < 0.001). There were remarkable differences between the MS and non-MS groups with regard to BMI, waist circumference, negative subscale of the PANSS scale, FPG, TG, and HDL-C (all *p* < 0.05). Elevated levels of Hcy, MIF, and hs-CRP were detected in the MS group compared to the non-MS group (all *p* < 0.05).

RETRACTED

**Conclusion:**

These findings suggest that increased concentrations of HCY, MIF, and hs-CRP may contribute to the abnormal glycolipid metabolism in the context of schizophrenia.

## 1. Introduction 

Schizophrenia is considered as a heterogeneous mental disease that is characterized by positive symptoms, such as hallucinations and delusions, and negative symptoms, including social withdrawal, depression, and a lack of motivation [1]. In addition, schizophrenia is related to cognitive impairment as well, such as executive function, memory, and mental processing speed [2, 3]. Some patients with schizophrenia are associated with symptoms of acute agitation and aggression, with the result of potential harm to themselves, peers, and healthcare workers [4]. The initial symptoms of schizophrenia usually are found in the late adolescence and early 20 s, and these children who later suffer from schizophrenia tend to have social disorders and mental retardation compared with their siblings of the same age [3]. Genetic factors related with the immune system and cytoskeleton, as well as environmental factors involving obstetrical complications, childhood trauma, and urban lifestyle, are contributed to the incidence of schizophrenia [5]. The Global Burden of Diseases Study reported that schizophrenia, as one of top 10 global causes of disabilities, was associated with nearly 1% population worldwide, which caused huge costs to the healthcare system [6, 7]. Schizophrenia is not only related to less daily activities and impaired physical health but also contributed to a reduced life expectancy (about 20 years) compared with the general population [8]. According to some research studies, the health-related risk factors involving cardiovascular diseases and metabolic abnormalities, such as hypertension, hyperlipidemia, and hyperglycemia, might be responsible for its high mortality [9], and compared with general population, the patients with schizophrenia are more prone to metabolic abnormalities and cardiovascular diseases, such as stroke and coronary heart disease [10, 11]. Additionally, it was found that about 37.3% of schizophrenic patients receiving second-generation antipsychotic drugs had metabolic abnormalities, which leaded to the risk of coronary heart disease [12], and it was more prevalent in schizophrenic patients with negative symptoms, related to sedentary lifestyle and less physical activity [13]. Therefore, the investigation of the glycolipid metabolism in schizophrenic patients is worth further exploring. In this study, we aimed at comparing the glycolipid metabolism in patients with first-episode schizophrenia (FES) with sex- and age-matched healthy controls to investigate changes in serum levels of homocysteine (Hcy), macrophage migration inhibitory factor (MIF), and high-sensitive C-reactive protein (hs-CRP) and their relationships with the glycolipid metabolism in patients with FES.

RETRACTED

## 2. Materials and Methods

### 2.1. Study Participants

Using a case-control design, 91 patients with schizophrenia were recruited from our hospital between January 2019 and May 2020. Inclusion criteria were initial diagnosis and second diagnosis after 4 weeks of first-episode schizophrenia by two trained psychiatrists using the Chinese Classification of Mental Disorders (CCMD-III), aged 18–60 years, Han Chinese, total scores on the Positive and Negative Syndrome Scale (PANSS) ≥60 (at least 3 items of the positive syndrome scale reaching 4 points or more), scores on the Young Mania Rating Scale (YMRS) <6, scores on the 17-item Hamilton Rating Scale for Depression (HAMD-17) <7, and informed of study objective and design. Each subject underwent a complete medical history, physical examination, and laboratory tests. Subjects with major medical abnormalities were excluded, including acute or unstable medical illnesses, suicide attempts, or any organic brain diseases. In addition, subjects suffering from drug or alcohol abuse/dependence and administrated with antipsychotics, antidepressants, or mood stabilizers in recent one month were excluded. Pregnant and lactating women were also excluded. The trained research staff collected general information and social-demographic characteristics through self-made questionnaires. Other information, including a history of mental illness and medications, were collected from medical records. Healthy controls (*n* = 88) were those who had received physical examinations at the same period, without the history or family history of mental illness.

### 2.2. PANSS, Personal and Social Performance (PSP) Scale, YMRS, HAMD-17, and Nottingham Onset Schedule (NOS)

The PANSS (interrater reliability at 75% among raters) [14] was used to assess the psychiatric symptoms of included patients, and the assessments were performed by two psychiatrists who had received same training skills to ensure consistency. There are 30 psychiatric parameters assessed on the PANSS including three subscales, a positive scale with 7 positive symptoms (*P*1–*P*7), a negative scale with 7 negative symptoms (*N*1–*N*7), and a general psychopathology scale with 16 items (*G*1–*G*16). Subscale scores were shown to be independent of each other, representing increasing levels of psychopathology severity. The PANSS is scored by summation of ratings across items, such that the positive and negative scales are scored with the potential range from 7 to 49, and the general psychopathology scale is scored with the potential range from 16 to 112. The PSP scale [15] is developed based on the social functioning component of the DSM-IV Social and Occupational Functioning Assessment Scale (SOFAS) as an instrument to assess social functioning in schizophrenia. Higher scores suggest better personal and social functioning, with score ranging from 91 to 100 reflecting more than adequate functioning, while scores <30 indicate so poor functioning that intensive supervision is required. The YMRS scale was employed to assess the severity of mania [16], which is an 11-item rating scale among which items 1–4, 7, 10, and 11 have a potential range from 0 to 4 for each, and items 5, 6, 8, and 9 have a potential range from 0 to 8 for each. Higher scores suggest severe mania. The HAMD-17 [17] scale was adopted to evaluate depressive symptoms, among which most of items have a potential range from 0 to 4 for each, and several items have a potential range from 0 to 2 for each. Higher scores suggest severe depression. The NOS is a short, guided interview and rating schedule to measure onset in psychosis [18], which is adopted to evaluate duration of untreated psychosis (DUP) and duration of untreated illness (DUI). DUP and DUI are defined as the time between the first ever onset of any psychiatric symptoms to the time of antipsychotic treatments.

RETRACTED

### 2.3. Glycolipid Metabolism

Measurements of the glycolipid metabolism comprised data from body mass index (BMI), waist circumference, blood pressure (BP), levels of fasting plasma glucose (FPG), 2-h glucose, fasting plasma insulin (FPI), impaired glucose tolerance (IGT), homeostasis model assessment of insulin resistance (HOMA2-IR), total cholesterol (TC), triglyceride (TG), low-density lipoprotein-cholesterol (LDL-C), and high-density lipoprotein-cholesterol (HDL-C). PBMI (weight (kg)/height squared (m^2^)) was calculated in a standardized fashion by assessing bodyweight and height. Weight was measured by a 0.1 kg electronic scale when the subjects wore light indoor clothing. Height was measured when the subjects stand upright on the floor of the height meter, with the heel close together, the tip toe of the foot is 60 degrees, the arms naturally droop, and the eyes are looking at the front horizontally. Venous blood (5 ml) was collected from each subject fasting for at least 8 hours and then centrifuged at 3000 r/min for 10 minutes within 30 min of collection. The serum and plasma were, respectively, isolated and stored at −80°C for testing. The levels of FPG, TG, TC, HDL-C, and LDL-C were measured by the Hitachi 7180 automatic analyzer (Hitachi, Japan). All biochemical analyses were performed by a technician in the clinical laboratory center of the hospital, who was blind to the status of subjects. After collection of fasting blood, the oral glucose tolerance test (OGTT) was performed. In brief, the patients were required to drink 75 g glucose dissolved in 300 ml water within 5 min, and blood samples were collected at 0.5, 1, 1.5, and 2 h for measurement of FPI. HOMA2-IR is used to estimate insulin resistance and was calculated using the equation HOMA-IR = FPI (IU/ml) × FPG (mmol/l)/22.5 [19].

### 2.4. Hcy, MIF, and hs-CRP Measurements

The levels of Hcy, MIF, and hs-CRP in the serum of patients were measured by enzyme linked immunosorbent assay (ELISA) using commercially available kits (Beijing Leadman Biotechnology Co., Ltd., China) and by the Hitachi 7180 automatic analyzer.

### 2.5. Statistical Analysis

Continuous variables were represented as means and standard deviations, and Student's *t*-test was employed for their group comparison. Categorical variables are expressed as proportions, and the chi-square test or Fisher's exact probability method was employed for their group comparison. Spearman correlation was used to assess the relationship between variables. Data management and analysis were performed with the use of SPSS22.0 software (IBM, USA). *P* < 0.05 was used to reflect statistical significance.

## 3. Results

### 3.1. Sociodemographic Characteristics

A total of 91 patients with FES were retrospectively analyzed. Following 4 weeks, it was found by reexamination that there was a case of mental disorder due to intracranial infection, a case of manic episode, and a case of delusional disorder. Ultimately, 88 eligible patients with first-episode schizophrenia were included in this study, and their blood samples were analyzed. The study design is shown in Figure 1. Demographics characteristics of study subjects by group are presented in Table 1. There was no significant difference in demographic and clinical characteristics between the patients with FES and healthy controls (all *p* > 0.05), except for the education level, BMI, and waist circumference. As given in Table 1, it was found that more FES patients had ≤9 years of education and fewer had >12 years of education than healthy controls (*p* < 0.05). The patients with FES exhibited a higher BMI than healthy controls (*p*=0.016). The waist circumference was enlarged in the patients with FES compared to healthy controls (both *p* < 0.001).

RETRACTED

### 3.2. Abnormal Glycolipid Metabolism in Patients with FES

Accumulating evidence shows that the abnormal glycolipid metabolism may be associated with schizophrenia. The patients with FES had a higher level of FPG than healthy controls (*p*=0.001), and the proportion of the high FPG level (FPG ≥ 6.1 mmol/L) was higher in patients with FES than healthy controls (*p* < 0.001). The level of blood glucose at OGTT2 (2-h glucose) was higher in patients with FES than healthy controls (*p* < 0.001). The proportion of IGT (blood glucose at OGTT2 ≥ 7.8 mmol/L) and the HOMA2-IR was both higher in patients with FES than healthy controls (*p* < 0.001). In addition, we found that the patients with FES presented a higher level of TG concomitant with a lower level of HDL-C than healthy controls (both *p* < 0.001). The data are detailed in Table 2.

### 3.3. Increased Serum Levels of Hcy, MIF, and hs-CRP in Patients with FES

Fasting venous blood was collected from patients with FES and healthy controls, and the serum was extracted to determine the levels of Hcy, MIF, and hs-CRP. It was revealed that the patients with FES showed higher serum levels of Hcy, MIF, and hs-CRP than healthy controls (all *p* < 0.001, Figure 2). When assessing the relationships between the levels of Hcy, MIF, and hs-CRP and clinical characteristics of patients with FES, results showed that the serum level of Hcy was highly positively correlated with the score of PANSS totals (*r* = 0.551) and the negative syndrome of the PANSS scale (*r* = 0.494). The serum levels of MIF and hs-CRP were only positively correlated with the negative syndrome of the PANSS scale (*r* = 0.320 and *r* = 0.446).

### 3.4. The Serum Levels of Hcy, MIF, and hs-CRP Were Correlated with Glycolipid Metabolism in Patients with FES

Since the glycolipid metabolism and elevated levels of Hcy, MIF, and hs-CRP are associated with schizophrenia, we are interested in the relationship between the levels of Hcy, MIF, hs-CRP and glycolipid metabolism in schizophrenia. As shown in Figure 3, the level of Hcy shared positive correlations with the levels of FPG, 2-h glucose, and HOMA2-IR; the level of MIF was only positively correlated with the level of HOMA2-IR; the level of hs-CRP had a positive correlation with both levels of FPG and 2-h glucose (all *p* < 0.001). As shown in Figure 4, the levels of Hcy, MIF, and hs-CRP all shared positive correlations with the TG level and negative correlations with the HDL-C level (all *p* < 0.001).

RETRACTED

### 3.5. The Serum Levels of Hcy, MIF, and hs-CRP in FES Patients with or without MS

To further verify the relationship between the levels of Hcy, MIF, hs-CRP and glycolipid metabolism in schizophrenia, patients with FES were classified into MS and non-MS groups according to three (or more) of the following diagnostic criteria: waist circumference more than 102 cm for male and 88 for female; SBP equal to and more than 130 mmHg (1 mmHg = 0.133 kPa) or DBP equal to and more than 85 mmHg; TG equal to and higher than 1.7 mmol/L (150 mg/dl); HDL-C lower than 1.03 mmol/L (40 mg/dl) for male and 1.29 mmol/L (50 mg/dl) for female; and FPG equal to and higher than 6.1 mmol/L. The MS and non-MS groups exhibited no significant difference in terms of gender, age, DUP, DUI, PANSS scale, PSP scale, SBP, and DBP (all *p* > 0.05). There were remarkable differences between the MS and non-MS groups with regard to BMI, waist circumference, negative subscale of the PANSS scale, FPG, TG, and HDL-C (all *p* < 0.05). Elevated levels of Hcy, MIF, and hs-CRP were detected in the MS group compared to the non-MS group (all *p* < 0.05). These results suggest that the levels of Hcy, MIF, and hs-CRP are associated with the presence of MS in schizophrenia, and MS may exert therapeutic implications in schizophrenia. The data are detailed in Table 3.

## 4. Discussion

Schizophrenia, as a complex and serious mental disease, which seems to be rooted in the destruction of brain development by heredity and environment, has a profound impact on individuals and society [20]. Schizophrenia is featured with progressive cognitive impairment in attention, working memory, and executive function, which usually occurs in late adolescence or early adulthood [21]. The prevalence of schizophrenia is relatively low, but it was associated with high rate of disability, which ranked 12^th^ in 310 diseases and injuries worldwide reported in 2016 [22]. In addition, people with schizophrenia are contributed to reduced life expectancy over time than those without the disease [23]. A possible explanation for the difference in mortality is the increased risk of metabolic abnormalities in schizophrenia, such as diabetes, obesity, hypertension, and hypercholesterolemia [24].

In this study, 88 cases of FES patients were selected as study subjects, in whom the serum levels of HCY, MIF, and hs-CRP were detected, so as to explore the correlation between the serum levels and glycolipid metabolism. According to the baseline data, it was found that a slight difference was observed in the demographic and clinical characteristics between the patients with FES and healthy controls, but the FES patients revealed lower education level, higher BIM, and larger waist circumference compared with healthy controls. Some researchers have indicated that the schizophrenic patients suffered from weight gain and waist circumference enlargement due to less physical activities and second-generation antipsychotics drugs [25].

RETRACTED

The study pointed out that compared with healthy controls, the FES patients were with higher FPG level and 2-hour PBG level, as well as higher HOMA2-IR value. In addition, there were more FES patients prone to obtain IGT, higher TG value, and lower HDL-C level. These evidences indicated that the FES patients were more likely to run the risk of diabetes and cardiovascular disease. The analysis we observed was similar to other studies, which suggested that the prevalence of type 2 diabetes in schizophrenia is 2–5 times higher than that in the general population [26]. More evidences showed that the increased TG was revealed as a biomarker of cardiovascular risk [27], and the lower HDL-C level influenced the efficacy of cardiovascular disease [28]; moreover, the schizophrenia was associated closely with short average life expectancy mostly due to cardiovascular deaths [29].

According to the serum data compared with healthy person, it was observed that the higher serum levels of Hcy, MIF, and hs-CRP were revealed in patients with FES. The Hcy level was significantly positively related with the PANSS scores and negative syndrome scale (PANSS), but the MIF and hs-CRP levels were positively correlated with negative syndrome scale (PANSS). The Hcy is thought to be a kind of nonprotein amino acids, and its increase is correlated with various diseases, such as heart and brain diseases, stroke, neurodegenerative diseases, diabetes, megaloblastic anemia [30], and even cancer risk factors [31]. MIF is one of the earliest inflammatory cytokines with unique structural characteristics, which was initially mentioned as a soluble factor produced by human lymphocyte in 1966 [32], and it is related to upregulation of immune responses and participation in the pathogenesis of autoimmune diseases [33]. Several studies have showed that the increased MIF expression was positively correlated with the dose of antipsychotic drugs, and it has been reported in patients with obesity or type 2 diabetes [34]. The CRP is considered as a conserved inflammatory plasma protein in the acute stage. In 1930, Tillet and Francis first discovered it when they studied the serum of patients with acute pneumococcal infection [35]. The hs-CRP concentration was contributed to the potential diagnosis for cardiovascular diseases since 2010 [36], and its increased concentration was approved to be associated with prediction of mortality in type 2 diabetes [37]. In this study, it was manifested that there were significant positive correlations between the Hcy level and FPG, PBG, and HOMA2-IR, and the MIF concentration was positively correlated with HOMA2-IR only. Additionally, it was indicated that the elevated levels of FPG and 2-hour PBG were relevant with increased hs-CRP concentration. Moreover, the Hcy, MIF, and hs-CRP levels were in positive correlation with the TG level, but with negative correlation to the HDL-C level. According to further detailed research data, which came from the FES patients in the MS and non-MS groups, it found a slight difference in the gender, age, DUP, DUI, PANSS scale, PSP scale, SBP, and DBP between the two groups. However, compared with the non-MS group, the FES patients in the MS group demonstrated a higher value of BMI, waist circumference, FPG, and TG and a lower level of HDL-C. There were more MS patients who tend to have negative symptoms of schizophrenia. In addition, the level of Hcy, MIF, and hs-CRP was higher in the MS group than that in the non-MS group. All the further verifications showed that the prevalence of MS significantly was associated with the Hcy, MIF, and hs-CRP concentration in patients with schizophrenia.

RETRACTED

Taken together, the serum levels of Hcy, MIF, and hs-CRP were significantly associated with the glycolipid metabolism in FES patients. The levels of Hcy, MIF, and hs-CRP were positively correlated with the TG level and negative correlations with the HDL-C level, and the elevated concentrations of Hcy, MIF, and hs-CRP were contributed to the metabolism abnormalities, which leaded to obesity, diabetes, and cardiovascular diseases. However, there was weak correlation between Hcy, MIF, and hs-CRP and the glycolipid metabolism in view of *r* values. Considering the relative sample size in this study, further investigations with larger sample population should be recruited. The data obtained from this study provide a better assessment of metabolic risk and indirectly predict the mortality caused by metabolism abnormalities in schizophrenia.

## Figures and Tables

**Figure 1:** Flow diagram of study design.

**Figure 2:** The serum levels of Hcy, MIF, and hs-CRP in patients with FES and healthy controls.

**Figure 3:** The relationship between the levels of Hcy, MIF, hs-CRP, and glycometabolism in patients with FES.

**Figure 4:** The relationship between the levels of Hcy, MIF, hs-CRP, and lipometabolism in patients with FES.

**Table 1:** Sociodemographics and clinical characteristics of patients with FES and healthy controls.

Characteristics	FES (*n* = 88)	Healthy controls (*n* = 88)	*P* value
Age (year)	24.56 ± 6.23	23.92 ± 5.33	0.465
Gender (male, %)	54 (61.36%)	49 (55.68%)	0.541

Living status (%)			
Married or cohabiting	17 (19.32%)	19 (21.59%)	0.709
Living with parents	45 (51.14%)	41 (46.59%)	0.546
Living alone	26 (29.54%)	28 (31.82%)	0.744

Education level (%)			
≤9	24 (27.27%)	11 (12.50%)	**0.014**
>9 and ≤ 12	43 (48.86%)	44 (50.00%)	0.880
>12	21 (23.86%)	33 (37.50%)	**0.049**
BMI (kg/m^2^)	24.72 ± 4.35	22.19 ± 3.98	**0.009**
Current smoking	20 (22.73%)	19 (21.59%)	0.856
Waist circumference (cm)	87.57 ± 6.26	72.22 ± 5.94	**<0.001**
SBP (mmHg)	120.30 ± 21.74	115.25 ± 20.66	0.116
DBP (mmHg)	82.08 ± 11.06	79.44 ± 9.23	0.087

The bold values indicate the comparison between the two groups is statistically significant.

RETRACTED

**Table 2:** The glycolipid metabolism in patients with FES and healthy controls.

Clinical variables	FES (*n* = 88)	Healthy controls (*n* = 88)	*P* value
FPG (mmol/L)	5.11 ± 0.93	4.75 ± 0.41	**0.001**
FPG ≥ 6.1 mmol/L (%)	15 (17.05%)	0 (%)	**<0.001**
2-Hour glucose (mmol/L)	6.36 ± 1.51	5.10 ± 0.89	**<0.001**
IGT (%)	21 (23.86%)	0 (%)	**<0.001**
HOMA2-IR	2.69 ± 0.59	1.61 ± 0.47	**<0.001**
TC (mmol/L)	5.09 ± 0.76	5.16 ± 0.82	0.764
TG (mmol/L)	1.86 ± 0.76	0.96 ± 0.35	**<0.001**
LDL-C (mmol/L)	2.28 ± 0.68	2.61 ± 0.57	0.314
HDL-C (mmol/L)	1.42 ± 0.22	1.59 ± 0.24	**<0.001**

**Table 3:** The relationships between the levels of Hcy, MIF, and hs-CRP and clinical characteristics of patients with FES.

Clinical variables	MS (*n* = 27)	Non-MS (*n* = 61)	*P* value
Age (year)	25.77 ± 6.68	24.10 ± 5.93	0.245
Gender (male, %)	15 (55.55%)	39 (63.93%)	0.484
DUP (week)	93.67 ± 124.72	85.48 ± 113.11	0.762
DUI (week)	297.55 ± 201.39	274.92 ± 176.43	0.597
Positive syndrome	16.54 ± 6.24	15.77 ± 5.11	0.249
Negative syndrome	18.38 ± 5.62	16.15 ± 4.01	**0.037**
General psychopathology	35.78 ± 9.33	33.53 ± 8.76	0.279
PANSS totals	70.70 ± 18.19	65.45 ± 13.88	0.142
PSP totals	60.73 ± 6.24	62.94 ± 6.79	0.153
BMI (kg/m^2^)	26.53 ± 5.08	23.24 ± 4.39	**0.003**
Waist circumference (cm)	89.78 ± 6.49	85.75 ± 6.72	**0.010**
SBP (mmHg)	124.33 ± 20.06	118.56 ± 19.13	0.202
DBP (mmHg)	84.18 ± 13.20	80.49 ± 12.65	0.216
FPG (mmol/L)	5.82 ± 0.77	4.87 ± 0.59	**<0.001**
TG (mmol/L)	2.12 ± 0.59	1.71 ± 0.63	**0.005**
HDL-C (mmol/L)	1.29 ± 0.18	1.48 ± 0.23	**<0.001**
Hcy (*μ*mol/L)	20.48 ± 5.03	17.59 ± 4.36	**0.008**
MIF (*μ*g/L)	54.63 ± 16.33	46.96 ± 15.39	**0.037**
hs-CRP (mg/L)	9.86 ± 2.64	8.37 ± 2.57	**0.015**

The bold indicate the comparison between the two groups is statistically significant.

## Data Availability

The data used to support the findings of this study are included within the article.
